# Clinical Significance of Neuregulin 4, Afamin, and SERPINB1 in Gestational Diabetes Mellitus and Their Relationship with Insulin Resistance

**DOI:** 10.1155/2022/2829662

**Published:** 2022-08-28

**Authors:** Qian Li, Chunmei Li, Jing Jin, Yang Shen, Mei Wang

**Affiliations:** ^1^Department of Obstetrics and Gynecology, Dongxihu People's Hospital, Wuhan, China; ^2^Endocrine Department, Dongxihu People's Hospital, Wuhan, China

## Abstract

**Objective:**

This study aims to explore the serum levels of neuregulin 4 (NRG4), afamin (AFM), and serpin family B member 1 (SERPINB1) in gestational diabetes mellitus (GDM) patients and their relationship with insulin resistance.

**Method:**

Serum levels of AFM, SERPINB1, and NRG4 were measured in GDM (*n* = 58), and non-GDM women (*n* = 60) using enzyme-linked immunosorbent assay (ELISA) kits. Besides, the serum insulin and glucose levels were also measured followed by calculating the homeostatic model assessment of insulin resistance (HOMA-IR). The correlation was performed using the Pearson analysis.

**Results:**

The increased serum levels of AFM and SERPINB1 were revealed in GDM patients as compared with non-GDM women, accompanied by the lower NRG4 serum level. ROCs for AFM concentrations showed an AUC of 0.629 (95% CI: 0.527∼0.731), 0.832 (95% CI: 0.754∼0.909) for the SERPINB1 serum level, and 0.626 (95% CI: 0.524∼0.728) for the NRG4 serum level. The threshold was 108.05 mg/L, 8.75 ng/mL, and 96.25 ng/mL of AFM, SERPINB1, and NRG4. Moreover, the combined ROC of AFM, SERPINB1, and NRG4 serum levels showed higher sensitivity (72.41%) and specificity (85.00%) for the diagnosis of GDM (AUC = 0.839; 95% CI: 0.764∼0.913). In GDM patients, the Pearson analysis revealed a significant correlation between AFM and SERPINB1 (*r* = 0.776), AFM and NRG4 (*r* = −0.799), as well as SERPINB1 and NRG4 (*r* = −0.783). Moreover, AFM and SERPINB1 serum concentrations in GDM patients were positively related to insulin levels, fasting glucose levels, and HOMA-IR values. However, the SERPINB1 serum level was negatively correlated with serum insulin and glucose levels and HOMA-IR.

**Conclusion:**

Abnormal serum levels of NRG4, AFM, and SERPINB1, as highly sensitive diagnostic tools, are closely related to insulin resistance in GDM patients.

## 1. Introduction

As hyperglycemia and glucose intolerance are first recognized in the second or third trimester of pregnancy, gestational diabetes mellitus (GDM) is not attributable to previous diabetes, which can cause several risks for pregnant women and their fetus, including an increased risk of developing type 2 diabetes and other obesity-related disorders [1, 2]. Insulin resistance is an important physiological process essential during pregnancy to ensure sufficient fetal nutrition, and the physiological changes in insulin are excessive in women with GDM, usually as a result of *β*-cell impairment [2]. GDM complicates approximately 1∼14% of all pregnancies worldwide with higher rates in Asia [3]. In mainland China, the incidence of GDM is 14.8%, which is similar to the reported incidence of GDM in Hong Kong (14.4%) [4].

At present, blood glucose screening is the most common method for the diagnosis of GDM in the middle and late stages of pregnancy. However, once diagnosed, there is little time left to treat GDM, leading to a negative impact on the fetus. Therefore, the identification of biomarkers for diagnosis and appropriate treatment of GDM is crucial in preventing maternal and neonatal complications [5, 6]. Neuregulins (NRGs) family (NRG1-4) is a signal protein containing epidermal growth factor-like domains, acting on tyrosine kinase receptors of the ErbB family (ErbB1-4), which participates in a variety of biological processes by mediating cell-cell interactions [7], such as stimulation, proliferation, apoptosis, migration, and differentiation [8]. As ligands for receptor tyrosine kinases of the ErbB family, NRGs have been found to be involved in the development of nervous systems, such as schizophrenia [9], organ systems such as heart and breast [10], and human diseases such as diverse cancers [11]. Neuregulin 4 (NRG4) is a specific ligand of ErbB4 and is mainly expressed and secreted by brown adipocytes [12]. Brown adipose tissue maintained body temperature higher than ambient temperatures and its activation alleviated obesity, with approximately 2.5–5% of contribution rate to human resting metabolic rate [13, 14]. As an 87,000-dalton protein, afamin (AFM) is a novel human serum protein that belongs to the albumin family localized on chromosome 4 and has specific binding properties for vitamin E [15]. An increased level of AFM was observed during persistent pregnancy secondary to hormonal changes [16]. It has been shown to play a vital role in the prevalence and incidence of type 2 diabetes mellitus [17]. Currently, the generation of insulin-secreting cells from human pluripotent stem cells [17] or the promotion of pancreatic *β* cell proliferation [18] contributed to reversing diabetes. Pancreatic *β* cells in response to insulin resistance were partially mediated by liver-derived protein [19]. As a liver-derived secretory protein, SERPINB1 was reported to promote pancreatic *β*-cell proliferation [20].

In this retrospective study, we collected clinical data of 60 non-GDM and 58 GDM women, evaluated the maternal circulating levels of NRG4, AFM, and SERPINB1 during pregnancy in GDM, and identified their diagnostic values.

## 2. Methods and Materials

### 2.1. Study Participants

Overall, all women (*n* = 118) over 18 years of age underwent a 75 g oral glucose tolerance test (OGTT) [21] in the second trimester (24∼28 weeks), and all did not receive medications that interfered with glucose or lipid metabolism before blood sampling. According to the result of OGTT screening, GDM was diagnosed if the subjects had fasting glucose ≥5.1 mmol/L, 1-hour glucose ≥10.0 mmol/L, and/or 2-hour glucose ≥8.5 mmol/L. There were 58 pregnant women diagnosed with GDM and the other women were not diagnosed with GDM (*n* = 60). Maternal prepregnancy body mass index (BMI) was calculated as weight/height^2^ (kg/m^2^) [22]. The gestational age was calculated according to the date of the last trustworthy menstrual period, which was then confirmed by the earliest pregnancy scanning [23].

### 2.2. Sample Size

We calculated the sample size by the G^*∗*^ Power software (latest ver. 3.1.9.7) using *t* tests (means: the difference between two independent means) [24]. We input the *β*/*α* ratio, effect size, and total sample size for the two groups in the main window, and the result showed a power of 0.927.

### 2.3. Exclusion Criteria

Exclusion criteria were as follows: (1) multiple pregnancy; (2) pregestational diabetes; (3) preexisting glucose intolerance; (4) pregnancy-induced hypertensive disease; (5) parathyroid and bone metabolism abnormalities; (6) syphilis, Hepatitis B virus, or HIV carrier; (7) acute or chronic inflammation; (8) allergic diseases; (9) smoking, alcohol use, or drug use; (10) a history of fetal anomalies; (11) premature rupture of membranes; and (12) a history of insulin therapy.

### 2.4. Sample Collection

An overnight fasting venous blood sample was collected from all study participants through venipuncture. The serum was obtained by centrifugation (5000 rpm for 15 min), and its aliquots were frozen and kept at −80°C until analysis. The serum levels of glucose and insulin were assessed using a human glucose assay kit (Catalog No. KA0831, Bio-Techne China Co. Ltd. Shanghai, China) and a human Insulin Quantikine Enzyme-linked immunosorbent assay (ELISA) kit (DINS00, Bio-Techne China Co. Ltd. Shanghai, China). Homeostatic model assessment of insulin resistance (HOMA-IR) was calculated using the following formula: fasting glucose (mmol/L) × fasting insulin (IU/mL)/22.5 [25].

### 2.5. Detection of AFM, SERPINB1, and NRG4 Serum Levels

The serum level of NRG4 (Catalog No. ABIN6968855, Antibodies-online GmbH, Aachen, Germany), AFM (Catalog No. ABIN6730921, Antibodies-online GmbH, Aachen, Germany), and SERPINB1 (Catalog No. ABIN6959408, Antibodies-online GmbH, Aachen, Germany) was measured using human ELISA kits. The interassay and interassay CV%, standard curve range, and sensitivity are listed in Table 1.

### 2.6. Statistical Analysis

Statistical package program SPSS 20 (Armonk, NY: IBM Corp.) was used to interpret the data with *P* < 0.05 as statistically significant. After the assessment for normality of data distribution using the Shapiro–Wilk test (data not shown), all the continuous variables in our study with normal distribution expressed as mean ± SD were performed using Student's *t*-test. Correlations were analyzed by the Pearson analysis.

## 3. Result

### 3.1. Subject Baseline Characteristics

The characteristics of 60 non-GDM and 58 GDM women are summarized in Table 2. For both groups, average ages, gestational age, and BMI were similar, with a mean of 29.5 ± 2.27 years in non-GDM and 29.57 ± 2.94 years in GDM women (*P*=0.891), a mean of 26.05 ± 1.35 weeks in non-GDM and 25.78 ± 1.36 weeks in GDM cases (*P*=0.274), as well as an average of 24.95 ± 2.42 kg/m^2^ in non-GDM and 25.04 ± 2.15 kg/m^2^ in GDM subjects (*P*=0.831). Moreover, no significant difference was observed regarding to HbA1C% (*P*=0.399), SBP (*P*=0.486), DBP (*P*=0.975), gravidity (*P*=0.599), and parity (*P*=0.813), indicating the patients were compared. Besides, GDM women had significantly serum insulin and glucose levels and HOMA-IR compared with non-GDM women (all *P* < 0.05).

### 3.2. Comparison of AFM, SERPINB1, and NRG4 Serum Levels in GDM and Non-GDM Women

As illustrated in Figure 1, the increased serum levels of AFM (97.44 ± 42.83 vs. 78.62 ± 36.32 mg/L, *t* = 2.579, *P*=0.011) and SERPINB1 (12.16 ± 5.02 vs. 6.37 ± 2.89 ng/mL, *t* = 7.707, *P* < 0.001) in GDM patients as compared with non-GDM women. Besides, GDM patients had lower NRG4 serum level than the non-GDM cases (84.86 ± 33.33 vs. 102.00 ± 46.00 ng/mL, *t* = 2.311, *P*=0.023).

### 3.3. The Diagnostic Effect of AFM, SERPINB1, and NRG4 Serum Levels in GDM

ROCs for AFM concentrations showed an AUC of 0.629 (95% CI: 0.527∼0.731, Figure 2(a)), 0.832 (95% CI: 0.754∼0.909, Figure 2(b)) for the SERPINB1 serum level, and 0.626 (95% CI: 0.524∼0.728, Figure 2(c)) for the NRG4 serum level. The threshold of AFM, SERPINB1, and NRG4 were 108.05 mg/L, 8.75 ng/mL, and 96.25 ng/mL, respectively, for distinguishing between women who developed GDM, and those who did not with the sensitivity of 44.38%, 75.86%, and 66.67%, as well as the specificity of 85.00%, 81.67%, and 62.07% (Table 3). Moreover, the combined ROC of AFM, SERPINB1, and NRG4 serum levels showed higher sensitivity (72.41%) and specificity (85.00%) for the diagnosis of GDM (AUC = 0.839; 95% CI: 0.764∼0.913, Figure 2(d), Table 3).

### 3.4. Correlation among AFM, SERPINB1, and NRG4 Serum Levels in GDM

To find the correlation among AFM, SERPINB1, and NRG4 serum levels in GDM, the Pearson analysis was then performed, and the result revealed a significant correlation between AFM and SERPINB1 (*r* = 0.776, *P* < 0.001), AFM and NRG4 (*r* = −0.799, *P* < 0.001), as well as SERPINB1 and NRG4 (*r* = −0.783, *P* < 0.001) in serum of GDM patients (Figure 3).

### 3.5. Correlation between AFM, SERPINB1, and NRG4 Serum Levels and Insulin Resistance

Moreover, AFM and SERPINB1 serum concentrations in GDM patients were positively related to insulin levels, fasting glucose levels, and HOMA-IR values (all *P* < 0.05). In terms of the NRG4 serum level, it was shown to be negatively correlated with serum insulin and glucose levels and HOMA-IR (all *P* < 0.05, Figure 4, Table 4).

## 4. Discussion

Women with GDM run a higher risk of developing maternal and perinatal complications including preeclampsia [26], type 2 diabetes mellitus after delivery [27], hypertension, and cardiovascular disease [28], and their infants are more likely to have adverse outcomes, such as neonatal hypoglycemia and polycythemia [29]. Therefore, a novel diagnosis for GDM is extremely important for the health of pregnant women and their fetuses.

AFM is a vitamin E-binding protein mainly secreted by the liver and exhibited antioxidant properties against related injuries and disease [30]. AFM has been reported to be increased in maternal serum during pregnancy and related to pregnancy-related complications. A pilot study presented by Hubalek et al. [31] revealed that in the first trimester, pregnant women with preeclampsia showed significantly higher median serum concentrations of AFM than that in pregnant healthy controls. Another study also indicated that compared to healthy pregnant women, elevated first-trimester serum AFM levels were observed in pregnant women with preeclampsia and GDM [32]. In our study, we included a total of 118 pregnant women consisting of GDM women and non-GDM women, and they were between 24 and 28 weeks of gestation (second trimester). The serum levels of AFM, SERPINB1, and NRG4 were determined, and it was observed that GDM patients revealed significantly higher serum levels of AFM than that non-GDM patients. Our results were a little different from another study, which suggested no significant difference in third-trimester AFM levels between GDM and non-GDM groups was discovered [33]. Furthermore, we performed ROCs to predict if AFM can be used as an indicator for GDM diagnosis, and the data showed AFM was with AUC of 0.629 (95% CI: 0.527∼0.731), specificity of 85.00%, and 108.05 mg/L as the threshold for distinguishing GDM patients from non-GDM patients. During pregnancy, the risk of pregnancy complications including GDM is associated with insulin resistance and insulin secretion [34]. Biochemical variables were evaluated in our study in response to the correlation between these and AFM, and we discovered that serum AFM level was significantly positively related to insulin levels, fasting glucose levels, and HOMA-IR values. Although there was no direct evidence supporting our above finding, other GDM studies confirmed that significantly higher levels of fasting blood glucose, fasting insulin, and HOMA-IR were revealed in pregnant women with GDM than that in controls [25]. Akbas et al. also demonstrated that these three biomarkers were increased in GDM patients compared to the controls, and serum cortistatin related to GDM was negatively correlated with these biomarkers [21].

NRG4 is a novel adipokine, which is primarily expressed in brown adipose tissue, and acts as a vital role in regulating metabolic homeostasis and maintaining energy. Previous evidence proved that NRG4 has been involved in several disorders related to obesity [35] and GDM [36]. Attique et al. concluded that NRG4 concentration declined in GDM females compared to the healthy group (*P* < 0.04) and showed a weak association with HOMA-IR but the significant inverse association with insulin, indicating a potential role of NRG4 in regulating insulin sensitivity, and its possibility as a biomarker of GDM [37]. During the second and third trimesters, Zhang et al. indicated the females in the control group exhibited significantly higher serum NRG4 concentration than the GDM females and NRG4 concentration was negatively related to fasting glucose and HOMA-IR [38]. These findings were similar to ours, which suggested that NRG4 expression decreased in GDM patients than that in non-GDM patients, and the difference was statistically significant. Moreover, there were negative relations between NRG4 levels and three biomarkers including insulin levels, fasting glucose levels, and HOMA-IR values. The ROCs data proved that NRG4, with an AUC of 0.626, a sensitivity of 66.67%, and a specificity of 62.07%, might be a potential biomarker of GDM diagnosis.

As a member of the clade B of SERPINS, the role of inflammation and cell migration of intracellular protein SERPINB1 has been widely explored [39, 40]. Recently, SERPINB1 has attracted attention in the treatment of diabetes mellitus treatment due to its role in inducing *β*-cell proliferation [41]. A small sample size of the study showed that elevated serum level of SERPINB1 was revealed in the patients with type 2 diabetes compared to the healthy controls, and SERPINB1 was significantly negatively correlated with serum low-density lipoprotein cholesterol [42]. In the present study, compared to non-GDM women, GDM women presented higher serum levels of SERPINB1. Furthermore, SERPINB1 showed an AUC of 0.832, a sensitivity of 75.86%, and a specificity of 81.67% for distinguishing between women with and without GDM. Kamal et al. demonstrated that higher SERPINB1 was associated with *β*-cell dysfunction and abnormal glycolipid, but no correlation was found between SERPINB1 and HOMA-IR both in non-type 2 diabetes and subjects with type 2 diabetes [41]. In our study, SERPINB1 serum concentration in GDM patients was positively related to insulin levels, fasting glucose levels, and HOMA-IR values.

In conclusion, our results show differences in the AFM, SERPINB1, and NRG4 serum levels between GDM and control pregnant group during pregnancy with high diagnostic values, which all were correlated with serum insulin and glucose levels and HOMA-IR.

To our knowledge, our study is one of the first to investigate the levels of the novel markers AFM, SERPINB1, and NRG4 in the GDM population. The combined ROC of AFM, SERPINB1, and NRG4 serum levels showed higher sensitivity and specificity for the diagnosis of GDM and provided a comprehensive overview of potential serum protein biomarkers for early GDM prediction.

However, a further study based on larger subjects is necessary to verify our results, and it still remains unclear whether these three serum levels can be used as biomarkers for the early screening of GDM. Moreover, the circulating concentrations in serum and plasma of AFM, SERPINB1, and NRG4 in different trimesters of pregnant women would be further explored in the future as time and funding permit.

## Figures and Tables

**Figure 1:** NRG4, AFM, and SERPINB1 serum levels were detected using ELISA. The increased serum levels of afamin (AFM, (a)) and serpin family B member 1 (SERPINB1, (b)) in gestational diabetes mellitus (GDM) patients as compared with non-GDM women accompanied by reduced neuregulin 4 (NRG4, (c)). ^*∗*^*P* < 0.05 and ^*∗∗∗∗*^*P* < 0.001 when compared to the non-GDM group.

**Figure 2:** The diagnostic effect of AFM, SERPINB1, and NRG4 serum levels in GDM. ROCs for afamin (AFM) concentrations showed an AUC of 0.629 (95% CI: 0.527∼0.731, (a)) of 0.832 (95% CI: 0.754∼0.909, (b)) for the serpin family B member 1 (SERPINB1) serum level, of 0.626 (95% CI: 0.524∼0.728, (c)) for the neuregulin 4 (NRG4) serum level, and of 0.839 (95% CI: 0.764∼0.913, (d)) for the combined detection of AFM, SERPINB1, and NRG4 serum levels.

**Figure 3:** Pearson analysis revealed a significant correlation between AFM and SERPINB1 (a), AFM and NRG4 (b), as well as SERPINB1 and NRG4 (c) in serum of GDM patients. Gestational diabetes mellitus (GDM), neuregulin 4 (NRG4), afamin (AFM), serpin family B member 1 (SERPINB1), and homeostatic model assessment of insulin resistance (HOMA-IR).

**Figure 4:** Correlations between AFM, SERPINB1, and NRG4 serum levels and insulin resistance in GDM patients. Gestational diabetes mellitus (GDM); neuregulin 4 (NRG4), afamin (AFM), serpin family B member 1 (SERPINB1), and homeostatic model assessment of insulin resistance (HOMA-IR).

**Table 1:** Detailed information on enzyme-linked immunosorbent assay (ELISA) kits.

Gene	Full names	Intra-assay CV%	Interassay CV%	Standard curve range	Sensitivity
NRG4	Neuregulin 4	<8	<10	0.781∼50 ng/mL	0.469 ng/mL
AFM	Afamin	<10	<12	3.12∼200 ng/mL	1.450 ng/mL
SERPINB1	Serpin family B member 1	<10	<12	0.31∼20 ng/mL	0.115 ng/mL

Neuregulin 4 (NRG4), afamin (AFM), serpin family B member 1 (SERPINB1), and coefficient of variation (CV).

**Table 2:** Demographic, clinical, and biochemical characteristics of study groups.

	GDM	Non-GDM	*t*	*P*
Age (years)	29.5 ± 2.27	29.57 ± 2.94	0.138	0.891
Gestational age (weeks)	25.78 ± 1.36	26.05 ± 1.35	1.099	0.274
BMI (kg/m^2^)	25.04 ± 2.15	24.95 ± 2.42	0.213	0.831
Newborn weight (g)	3.03 ± 0.53	2.9 ± 0.51	1.294	0.198
HbA1C%	5.00 ± 0.64	4.91 ± 0.56	0.847	0.399
SBP (mmHg)	106.4 ± 8.47	105.3 ± 9.80	0.700	0.486
DBP (mmHg)	74.53 ± 8.72	74.48 ± 8.72	0.032	0.975
Gravidity	2.14 ± 1.13	2.25 ± 1.17	0.528	0.599
Parity	0.98 ± 0.71	1.02 ± 0.83	0.237	0.813
Fasting glucose (mmol/L)	7.8 ± 1.15	7.08 ± 0.57	4.353	<0.001
Fasting insulin (IU/mL)	9.66 ± 4.36	8.29 ± 1.74	2.250	0.026
HOMA-IR	3.42 ± 1.72	2.61 ± 0.6	3.415	0.001

Gestational diabetes mellitus (GDM), body mass index (BMI), hemoglobin A1C (HbA1c), systolic blood pressure (SBP), diastolic blood pressure (DBP), and homeostatic model assessment of insulin resistance (HOMA-IR).

**Table 3:** Results of ROC analyses.

Parameter	AUC (95% CI)	Threshold	Sensitivity (%)	Specificity (%)
AFM	0.629 (0.527∼0.731)	108.05 mg/L	44.83	85.00
SERPINB1	0.832 (0.754∼0.909)	8.75 ng/mL	75.86	81.67
NRG4	0.626 (0.524∼0.728)	96.25 ng/mL	66.67	62.07
Combined	0.839 (0.764∼0.913)	0.538	72.41	85.00

Neuregulin 4 (NRG4), afamin (AFM), serpin family B member 1 (SERPINB1), receiver operating characteristic (ROC), and area under the ROC curve (AUC).

**Table 4:** Correlations between AFM, SERPINB1, and NRG4 serum levels and insulin resistance in GDM patients.

Parameter	*AFM (mg/L)*		*SERPINB1 (ng/mL)*		*NRG4 (ng/mL)*	
	*R*	*P*	*r*	*P*	*r*	*P*
Fasting glucose (mmol/L)	0.334	0.010	0.420	0.001	−0.432	0.001
Fasting insulin (IU/mL)	0.699	<0.001	0.727	<0.001	−0.755	<0.001
HOMA-IR	0.688	<0.001	0.737	<0.001	−0.773	<0.001

Neuregulin 4 (NRG4), afamin (AFM), serpin family B member 1 (SERPINB1), and homeostatic model assessment of insulin resistance (HOMA-IR).

## Data Availability

The data used to support the findings of this study are included in the article.
